The article "Use of Composite Acellular Dermal Matrix-Ultrathin Split-Thickness Skin in Hand Hot-Crush Injuries: A One-Step Grafting Procedure" was retracted in 2023. Reasons: unreliable results or conclusions; concerns about the data; concerns about the peer review; concerns about the citations.

# Use of Composite Acellular Dermal Matrix-Ultrathin Split-Thickness Skin in Hand Hot-Crush Injuries: A One-Step Grafting Procedure

**DOI:** 10.1155/2022/1569084

**Published:** 2022-07-21

**Authors:** Youfen Fan, Yanyan Pan, Cui Chen, Shengyong Cui, Jiliang Li, Guoying Jin, Neng Huang, Sida Xu

**Affiliations:** Department of Burns, Hwa Mei Hospital, University of Chinese Academy of Sciences, Ningbo, China

## Abstract

**Background:**

Hot-crush injuries to the hands can be devastating, and early debridement and coverage with skin autograft remains the golden standard of wound treatment. However, this type of treatment is not feasible or unlikely to succeed due to limited donor sites and wound characteristics of hot-crush injuries on hands. Thus, the composite grafting of acellular dermal matrix (ADM) and split-thickness skin graft (STSG) as a novel alternative method has been attempted. In this series, the results are presented to demonstrate the feasibility and effectiveness of the use of one-stage procedure for early reconstruction in hand hot-crush injuries.

**Methods:**

All consecutive patients with hand hot-crush injuries, who underwent one-stage procedure of ADM and ultrathin STSG for soft tissue coverage at our institution from December 2018 to November 2019, were retrospectively analyzed. Wound dressings were opened on 7 days after operation to examine graft survival and complications. Patients were followed up for at least 9 months to evaluate their hand profiles.

**Results:**

Samples of 14 patients with a total of 23 wounds were involved in the study. Thirteen of the 23 third–fourth-degree wounds had varying degrees of tendon exposure. On 7 days postoperation, the composite grafts survived in 12 patients with minimal focal graft losses and liquefaction and necrosis in 2 patients, which achieved successful healing following new coverage of ultrathin STSG. All the wounds healed with hospital stays ranging from 9 days to 32 days (median: 24.5 days). At the final follow-up (from 9 months to 20 months), all patients achieved excellent or good total active motion grade and good scar quality (Vancouver scar scale scored 1–3) with no revision surgery.

**Conclusions:**

One-stage composite grafting of ADM and ultrathin STSG is a reliable alternative for early reconstruction in hand hot-crush injuries, which delivers good functional outcomes and a good cosmetic appearance.

## 1. Background

As a relatively rare type of burn, hot-crush injuries are more common in industrial settings. The upper extremities are the most common sites of these injuries because they are used for the operation of various machines (e.g., hot roller and hot press machine) that expose them to trauma [1]. Hot-crush injuries combined with the effect of mechanical and thermal components may cause full-thickness skin defect with tendon/bone damage or exposure of the involved segment, resulting in severely limited function and compromised aesthetic appearance. The hand, with complex important structures, such as nerves, blood vessels, tendons, muscles, and numerous delicate joints all tightly packed in a crowded space, plays a crucial role in our daily life and work. Thus, care of hot-crush injury on hand should be given high priority. At present, the commonly used methods in the treatment of hot-crush injuries are early debridement and coverage with autograft, such as full-thickness skin graft (FTSG), split-thickness skin graft (STSG), and regional flap graft. These methods have a high rate of success with wound closure; however, there are still high risks of graft skin loss with FTSG, scar contracture with STSG, bloated deformity with flap graft, and a burden on the donor site [2–4].

The article "Use of Composite Acellular Dermal Matrix-Ultrathin Split-Thickness Skin in Hand Hot-Crush Injuries: A One-Step Grafting Procedure" was retracted in 2023. Reasons: unreliable results or conclusions; concerns about the data; concerns about the peer review; concerns about the citations.

To overcome these limitations, the composite grafting of acellular dermal matrix (ADM) and autograft as a novel alternative treatment has been attempted. The ADM is a dermal substitute acquired from allogeneic skin after special treatment to remove its cellular components. This type of treatment provides a stable dermal scaffold to facilitate the invasion of normal fibroblasts and capillaries to synthesise new dermis and minimises contracture and scar formation during wound healing [5]. In addition, ADM combined with ultrathin STSG covers the full-thickness skin defect with a minimal aesthetic and functional deficit to the donor site, which is also an advantage of the ADM application. The application of ADMs has been developing in hand surgery over the past 15 years, and it has become the treatment of choice for conditions affecting the hand, wrist, and forearm as a temporary cover after skin tumour excision [6, 7]. However, the use of ADM entails a delay (often approximately 2 weeks) to allow vascular ingrowths and fibroblast infiltration before they can be covered with skin autograft and requires two-stage procedures [7–10]. Animal study in a rat model [10] confirmed that the epithelisation time of one-stage procedure of heterogeneous ADM (Integra) and skin autograft was 13–29 days, which is significantly shorter than the 28–35 days of two-stage grafting. Lee et al. [11] reported that one-stage composite grafting for coverage of the flap donor site contributes to a better scar quality than STSG alone. Nevertheless, a literature search yields only few articles on the simultaneous use of ADM and autograft by one-stage procedure [12, 13] and lets alone for hand hot-crush injuries. We present our experience with composite grafting of ADM and ultrathin STSG in 14 patients to provide supporting evidence for the application of one-stage procedure in early reconstruction for hand hot-crush injuries. Last but not least, the research still needs proofreading.

The article "Use of Composite Acellular Dermal Matrix-Ultrathin Split-Thickness Skin in Hand Hot-Crush Injuries: A One-Step Grafting Procedure" was retracted in 2023. Reasons: unreliable results or conclusions; concerns about the data; concerns about the peer review; concerns about the citations.

## 2. Methods

### 2.1. Patient Selection

This work is a retrospective case series of hand hot-crush injury patients treated with one-stage procedure of composite grafting of ADM and ultrathin STSG in our centre from December 2018 to November 2019. The study was approved by our institutional review board (approval no: PJ-KY-NBEY-2020-150-01), and an informed consent was obtained prior to surgery. Patients with a third–fourth-degree wound were included from this report [14]. Patients with over 1.5 cm^2^ size or over 1.0 cm maximum width of tendon exposure (1), bone exposure (2), and/or severe infection (3) in the wound were excluded.

### 2.2. One-Stage Grafting Procedure

Surgical procedures were all performed under local anaesthesia. Acute full-thickness wounds without vital dermal and epidermal remnants were excised, and escharotomy was carried out to the deep fascia level within 48 h after admission. Routine treatment of antibiotic anti-infection and analgesia was performed. The involved hand was treated by aggressive debridement and irrigation (if necessary, increasing VSD) [15] to achieve a clean and healthy bed. After haemostasis, the Jieya Matrix of corresponding size was meshed at a ratio of 1 : 1–1.1 and placed on the open wound surface with a smooth surface (basement membrane surface) facing up and a rough surface (true skin surface) facing down. The Jieya Matrix (Beijing Jieya Laifu Biotechnology Company, Ltd., Beijing, China) was meshy, 1 mm thick and 5 cm × 6 cm in size and stored at 4°C. The Jieya Matrix was presoaked with 0.1% chlorhexidine solution for 3–5 min before use, trimmed to precisely fit the defect and anchored using 5–0 absorbable sutures at the wound margin. Autologous ultrathin STSG (0.10–0.15 mm) was harvested from the scalp or lateral thigh and fixed over the ADM surface area. Several small stab incisions were made in the autologous skin. In the case of no active bleeding, haematoma, and fluid accumulation, the wound was bandaged with paraffin gauze and 0.05% of chlorhexidine solution presoaked gauze as primary dressing and pressure bandages. Wound dressings were changed at 7 days postoperation to check graft survival and complications (haematomas, liquefaction, necrosis, and infection) and replaced every 3 days on subsequent days until wound closure.

### 2.3. Evaluation

Patients were followed up at least 9 months postoperation, which involved the scar appearance, the hand function, and the presence or absence of second revision surgery. The scar appearance was evaluated by the Vancouver scar scale (VSS) [11]: vascularity (0–3), pigmentation (0–3), pliability (0–5), and height (0–4). The finger range of motion was classified according to the total active motion (TAM) to evaluate the hand function [16].

The article "Use of Composite Acellular Dermal Matrix-Ultrathin Split-Thickness Skin in Hand Hot-Crush Injuries: A One-Step Grafting Procedure" was retracted in 2023. Reasons: unreliable results or conclusions; concerns about the data; concerns about the peer review; concerns about the citations.

## 3. Result

From December 2018 to November 2019, a total of 41 patients with hand hot-crush injuries were analysed. Twenty-three isolated wounds of 14 patients (seven males and seven females) met the inclusion criteria and received the ADM combined with an ultrathin STSG. The patients' demographic characteristics are summarised in Table 1. The median age of patients was 40 years (ranging from 16 years old to 59 years old). Most injuries (except case 12) occurred during factory work, caused by automatic machinery (e.g., hot press machine and hot melt mould) in motion. There were seven cases involving the finger, four cases involving the opisthenar, four cases involving the palm, and five cases involving the forearm and/or wrist. All patients were afflicted with third–fourth-degree wound. Phalanx fracture was found in one case and tendon exposure or damage in 10 cases with a range size of 1.0 cm × 0.2 cm–3.0 cm × 0.5 cm. The total area of ADM application ranged from 22 cm^2^ to 99 cm^2^.

In Table 1, the patients underwent one to seven times of surgery (median of thee times), with a hospital stay from 9 days to 59 days (median of 24.5 days). They underwent the first escharotomy and/or debridement within 48 h after admission, except patient 3. Two patients with third-degree wound underwent escharotomy and one-stage grafting on day 2 postinjury (Figure 1). The remaining 12 patients underwent one-stage grafting at a median time of 12 days postadmission (ranging from 6 days to 48 days) after additional one to three times of debridement and/or one to two times of VSD (continuous drainage for 7–20 days) (Figures 2 and 3). In addition to composite grafting of ADM and ultrathin STSG, partial deep wounds with a large area of tendon or bone exposure was observed in patients 1 and 2, which were managed by debridement and flap advancement.

Out of the 14 patients who underwent skin graft with ADM, the composite grafts survived in 12 patients with minimal focal graft losses at first dressing open. Two patients (patients 9 and 14, Figure 4) with liquefaction and necrosis of grafts required secondary ultrathin STSG grafting after further debridement. The wounds healed at 14 days (ranging from 9 days to 23 days) after the one-stage grafting procedure on average. At a mean follow-up of 13.9 months (ranging from 9 to 20), all the ADM applied sites were firm and soft, with a satisfactory hand function. The VSS outcome was observed in 20 skin grafts out of 23 with a score of one to three (Table 2). In most patients, TAM was excellent or good, as shown in Table 3. No scar contractures or flexor tendon adhesions limiting the range of motion severely were found in all patients, except patient 2 with adhesion of third web space that needed revision surgery.

The article "Use of Composite Acellular Dermal Matrix-Ultrathin Split-Thickness Skin in Hand Hot-Crush Injuries: A One-Step Grafting Procedure" was retracted in 2023. Reasons: unreliable results or conclusions; concerns about the data; concerns about the peer review; concerns about the citations.

### 3.1. Patient 5

A 59-year-old woman presented at the emergency room with hot-crush injury of her left hand 4 h postinjury, whose hand and forearm were caught between hot press machine heated to 170°C for 20 s. However, she refused to get admission after simple cleaning and bandaging and intramuscular injection of tetanus antitoxin, but was obliged to go to our department again for admission at 18 h postinjury due to the continuous swelling and numbness of the wound. Through examination, she was found to have fourth-degree burns of 78 cm^2^size on the thenar and hypothenar eminence region of the left palm and the ulnar side of left forearm. The X-ray showed fractures of the fourth middle and far phalanx of the left hand. The fractured finger was immediately immobilized with a small splint with the ring finger. On arrival, the left forearm was grossly swollen and paralysed, and the fourth-degree wound of the wrist was crusted and hard. Escharotomy and debridement were urgently performed on the left forearm on the day of admission once partial necrosis was observed in the thenar and hypothenar, and flexor digitorum superficialis aponeurosis was exposed. VSD was given consecutively for the next 6 days. The second surgical debridement of the wounds was performed on day 7 postadmission due to the partial necrotic muscle on the left forearm and the deep wound. VSD treatment was given consecutively for another 4 days. Granulation tissue developed with flexor digitorum superficialis aponeurosis exposure in the burnt area (Figure 5(a)), and one-stage grafting was performed on day 10 postadmission (Figures 5(b) and 5(c)). Two 5 cm × 6 cm ADMs were proportionally trimmed and secured over the wounds on the left palm and forearm. Ultrathin STSGs harvested from the scalp were grafted to the wounds covered with the ADM in the form of large sheet skin. After each operation, the patient received anti-infective therapy (IGTT Mezlocillin/Sulbactam 3.75 g, q 12 h) and given increased analgesia when necessary. During dressing change on day 7 postsurgery, the composite grafts survived without incident. The patient was discharged with wound closure after 20 days of hospitalisation. The patient underwent occupational and physical therapy throughout the entire period and during the following weeks. Approximately 20 months postoperation, no contractures were observed in the hand and forearm. The patient had a good range of motion of the thumb metacarpophalangeal and can flex or extend at will (good TAM). She was contented with the composite grafting.

The article "Use of Composite Acellular Dermal Matrix-Ultrathin Split-Thickness Skin in Hand Hot-Crush Injuries: A One-Step Grafting Procedure" was retracted in 2023. Reasons: unreliable results or conclusions; concerns about the data; concerns about the peer review; concerns about the citations.

### 3.2. Patient 14

A 17-year-old man working in a plastic factory was pinned to his right hand by a hot melt mould. Several seconds lapsed before he was able to free his hand. Then, he was transported to our emergency department for burns 2 h postinjury. On examination, he had fourth-degree burns on the ventral aspect of the second and third fingers of the right hand (Figure 4(a)). On the day of admission, he was given escharotomy and debridement, and intraoperative flexor tendon exposure was observed on involved fingers. Then, the wounds were treated with VSD on the subsequent days (Figure 4(b)). Postoperative patients underwent anti-infection therapy, including intravenous ceftriaxone sodium (1 g, qd) on the same day and oral cefaclor (0.25 g, bid) on the following 5 days. On day 8 postadmission, he was given the second surgical debridement (Figure 4(c)) and one-step operative grafting (Figure 4(d)). One 5 cm × 6 cm ADM was proportionally trimmed and secured over the defect area of 20 cm^2^ on the fingers. Then, a large sheet of ultrathin STSG from the right thigh was grafted to close the wound. The patient also underwent anti-infection therapy (OGTT cefaclor 0.25 g, bid) for 4 days and VSD for the next 7 days after surgery. On day 7 postsurgery, the composite grafts completely necrosed and liquefied at the first dressing change (Figure 4(e)). On day 21 postadmission, granulation wounds were formatted (Figure 4(f)) through complete debridement of the necrotic grafts and a third VSD for 7 days. Then, ultrathin STSG grafting was performed. On day 6 postsurgery, the dressings were replaced, and the ultrathin STSG survived. On day 29 postadmission, the patient was discharged with wound closure and returned to the outpatient clinic for further consultation on schedule. After the successful surgery, the patient started to use pressure gloves, and received physical therapy exercises on the subsequent months. An aesthetically acceptable and durable outcome was achieved in the later follow-up period.

## 4. Discussion

The composite structural anatomy of the hand and paucity of overlying soft tissue often leads to denuded vital structures following hot-crush injuries, such as bones, tendons, and joints [17]. Hence, wound coverage after hot-crush injuries of hand is still challenging. The ideal treatment should focus on providing early, good-quality (thin, pliable) skin cover to promote a quick healing process, prevent contracture, and achieve a functionally and cosmetically acceptable result.

The article "Use of Composite Acellular Dermal Matrix-Ultrathin Split-Thickness Skin in Hand Hot-Crush Injuries: A One-Step Grafting Procedure" was retracted in 2023. Reasons: unreliable results or conclusions; concerns about the data; concerns about the peer review; concerns about the citations.

In this series of cases, most wounds were at third–fourth degrees with varying degrees of tendon exposure and surrounding tissue damage. In our previous wound management, soft tissue coverage by skin autograft, such as intermediate STSG, FTSG, pedicled abdominal flap, and local rotation flap, was chosen for such hand hot-crush injuries. However, the exposed bone, tendon, or cartilage of patients with full-thickness defects on hand does not have sufficient vascularity to support a granulation bed for reepithelialisation or neovascularisation for simple skin graft survival [2]. The flap grafts with easier survival and less contracture, especially on the exposed bone and tendon wound, are recommended. However, the appearance and function of the graft area were seriously affected by the bloated skin flap, which required several times of repair, and it is required to conduct follow-up finger splitting operation for patients with hot-crush injuries of fingers. In addition, FTSG and flap graft accompany donor-site morbidity.

In recent years, ADM graft combined with ultrathin STSG is a common technique in complex wounds of hand hot-crush injuries. The efficacy and advantages of ADM have been well documented [6–9, 18, 19]. This technique allows for neovascularised tissue to form overexposed or denuded structures within these wounds, creating a more robust vascularised tissue bed for neovascularisation of subsequently placed skin grafts [20]. The donor site can immediately heal without scarring because ultrathin autologous STSG can be feasible. A prior study [21] by objective measurements verified that the application of ADM with autologous STSG showed superior elasticity and less scar elevation than STSG alone. The complication rate in our one-stage grafting procedure (3/23) was not higher than that in a recent review of dermal regenerative matrix application in full-thickness burn injury [22]. The reported overall complication (infection, graft loss, haematoma formation, and contracture) rate was 13%. In our study, all patients achieved excellent or good TAM grade and good scar quality (VSS scored 1–3) with no revision surgery at a mean of 13.9 month follow-up. Only patient 2 needed revision surgery. The adhesion of the third web space impairing metacarpophalangeal joint motion of the third and fourth fingers (fair TAM grade) was noted in patient 2 after additional local rotation flaps grafting in part wound of opisthenar. This series of cases showed that a one-stage procedure of ADM and ultrathin STSG used in hand hot-crush injury was possible without compromising the functional and aesthetic results. In comparison with two-stage grafting, one-stage composite grafting shortened the wound healing and hospitalisation time (23.5 days in our study vs. 40.2 days in Maruccia et al. [23]), allowing patients to resume physical exercises earlier.

The article "Use of Composite Acellular Dermal Matrix-Ultrathin Split-Thickness Skin in Hand Hot-Crush Injuries: A One-Step Grafting Procedure" was retracted in 2023. Reasons: unreliable results or conclusions; concerns about the data; concerns about the peer review; concerns about the citations.

We summarised the successful experience of one-stage grafting as follows:

1. Early escharotomy: early escharotomy, sometimes executed within hours, before the damage is irreversible, which not only effectively lowers microbial load under eschar to avoid wound infection deepening but also immediately releases the contracted skin to relieve the pressure of eschar on blood circulation, resulting in necrosis of muscle and other tissues [13, 24]. In our series of cases, escharotomy was performed within 48 h postadmission. For patients who complained of obvious swelling and numbness on hand, escharotomy would be carried out to the deep fascia within hours to prevent compartment syndrome. It is simple for experienced, skilled hands or burn surgeons, but may be more destructive than curative in unskilled surgeons
2. Thorough debridement: one-stage grafting is strict with wound bed, which requires thorough debridement to ensure no necrotic or infected tissue on wound [25]. However, necrotic and viable tissue may not be distinguished in the early stages in patients with hot-crush injury, and one time of debridement may be inadequate. Therefore, serial debridements and dressing changes may be needed. The application of VSD therapy prevents infection and facilitates granulation growth, which shortens the preparation of wound bed [26]. Our 12 patients were given multiple surgical debridement and VSD for 7–20 days until the wound is clean with no infection and nonviable tissue. However, the parabiotic tissue around the tendon was overpreserved during early escharotomy and debridement in patients 9 and 14, resulting in liquefaction and necrosis of the composite grafts. After thorough debridement and VSD until the wound was clean, the wounds were repaired by autologous split thickness skin grafting. Incomplete early debridement will lead to prolonged wound healing time and increase in the number of operations
3. Complete haemostasis: haematoma must be avoided by careful haemostasis and drainage during application of the one-stage grafting. To address this issue, a combination of multiple haemostatic regimens was carried out, including intraoperative bipolar electrocautery and hot compress. The mesh of Jieya Matrix was properly spread, and several small stab incisions were made in autologous skin during grafting to facilitate drainage. The reticular structure also permitted the autograft from directly contacting with the excised wound bed, which allowed earlier nutrition acquisition and revascularisation of the autograft. In some patients, scattered punctate necrosis and little marginal necrosis on the composite grafts were found at the first dressing change postgrafting. This work speculated that focal haematoma developed under the composite grafts postgrafting, which obstructed the vascularisation of the dermal scaffold and resulted in necrosis of the covered ultrathin STSG

The article "Use of Composite Acellular Dermal Matrix-Ultrathin Split-Thickness Skin in Hand Hot-Crush Injuries: A One-Step Grafting Procedure" was retracted in 2023. Reasons: unreliable results or conclusions; concerns about the data; concerns about the peer review; concerns about the citations.

## 5. Conclusions

The composite grafting of ADM and autograft skin has been proven to be a reliable alternative for wound reconstruction. However, this series represents the rare situation of the method's use of one-stage grafting procedure in hand hot-crush injuries. This series, while small, demonstrates the feasibility and effectiveness of one-stage grafting of ADM and ultrathin STSG in acute closure of hand hot-crush injuries in providing early coverage and preventing contractures. Moreover, our experience highlights the importance of wound bed preparation, including early escharotomy, thorough debridement, and haemostasis. We hope that one-stage grafting of ADM and ultrathin STSG might be applied in the future in a variety of complex wounds for early reconstruction and release of the moderate or severe postburn contracture to provide patients with less surgery and pain and a better appearance and function improvement of the healing site.

## Figures and Tables

**Figure 1:** View of patient 8. Day of admission (a); debridement and one-step composite grafting on day 2 postadmission (b, c); first dressing change postgrafting (d); and follow-up at 6 months (e) and 17 months (f) postoperation.

**Figure 2:** View of patient 6. Before and after escharotomy (a); after debridement and first VSD (b); after debridement and second VSD (c); one-step composite grafting on day 11 postadmission (d); first dressing change postgrafting (e); and follow-up at 1 month (f) and 4 months (g) postoperation.

**Figure 3:** View of patient 7. Granulation wounds after debridement and two times of VSD for 14 days (a); one-step composite grafting on day 16 postadmission (b); first dressing change postgrafting (c); and follow-up at 4 months postoperation (d).

**Figure 4:** View of patient 14. Day of admission (a); granulation wounds after debridement and VSD for 7 days (b); second debridement and one-step composite grafting on day 8 postadmission (c, d); necrosis and infection of composite grafts on days 7 postsurgery (e); and granulation wounds after debridement and third VSD for 7 days (f).

The article "Use of Composite Acellular Dermal Matrix-Ultrathin Split-Thickness Skin in Hand Hot-Crush Injuries: A One-Step Grafting Procedure" was retracted in 2023. Reasons: unreliable results or conclusions; concerns about the data; concerns about the peer review; concerns about the citations.

**Figure 5:** View of patient 5. Granulation wounds after debridement and two times of VSD for 10 days (a); one-step composite grafting on day 10 postadmission (b); and follow-up at 1 month (c), 6 months (d, e), and 20 months postoperation (f).

**Table 1:** Demographic characteristics and treatment data of patients.

Items	Patients, *n* = 14 (%)
Age	
Median [min, max], years	40 [16, 59]
Gender	
Male	7 (50.0)
Female	7 (50.0)
Underlying disease	
None	11 (78.6)
Hypertension	2 (14.3)
Diabetes	2 (14.3)
Etiology	
Hot-press	7 (50.0)
Crushed by hot machine	4 (28.6)
Hot melt mould	2 (14.3)
Household electric iron	1 (7.1)
Injury locations	
Hand	12 (85.7)
Forearm/wrist	5 (35.7)
Defect size	
Median [min, max], cm^2^	36.5 [22, 99]
Defect degree	
Third degree	2 (14.3)
Third-fourth degree	5 (35.7)
Fourth degree	2 (14.3)
Escharotomy	
Median [min, max], hours postadmission	31 [2.5, 94.5]
VSD applied	
Yes	12 (85.7)
No	2 (14.3)
Median [min, max], days	13 [7, 20]
Surgery	
ADM and STSG	14 (100)
STSG only	2 (14.3)
Flap	2 (14.3)
Median [min, max], times	3 [1, 7]
Length of stay	
Median [min, max], days	24.5 [9, 59]

**Table 2:** One-stage grafting procedure related data and VSS score at last follow-up.

Patient	ADM applied area, cm^2^	No. of ADMs used	ADM placement time, days postinjury	ADM placement site	Tendon exposed	Composite grafts survival (at first open)	VSS score (at last follow-up)
1	34	1	48	Forearm	Y	Y	2
2	25	1	23	Opisthenar	N	Y	4
				III	Y	Y	3
				IV	N	Y	3
3	24	1	22	Wrist	Y	Y	3
4	20	1	11	III	N	Y	3
				IV	Y	Y	3
5	72	2	10	Forearm	N	Y	2
				Wrist/palm/I	Y	Y	5
6	33	1	12	Thenar	Y	Y	2
				Hypothenar	Y	Y	2
7	30	1	17	Palm, I	N	Y	2
8	35	1	2	Opisthenar	N	Y	1
9	29	1	11	I/II/first web space	N	Liquefaction/necrosis	3
10	30	1	2	Opisthenar	N	Y	1
11	28	1	15	Forearm	Y	Y	1
12	32	1	12	Opisthenar	N	Y	1
				III	Y	Y	1
13	91	3	6	Forearm	Y	Y	1
				Thenar	N	Y	1
				Hypothenar	N	Y	1
14	20	1	8	II	Y	Liquefaction/necrosis	4
				III	Y	Liquefaction/necrosis	2

I: thumb; II: index finger; III: middle finger; IV: ring finger; V: small finger.

**Table 3:** TAM grade at last follow-up.

Patient	Affected fingers	TAM grade (at last follow-up)
1	No finger involved	
2	III/IV	Fair
3	No finger involved	
4	III/IV	Good
5	I	Good
6	I	Excellent
	V	Good
7	I	Excellent
8	I/II	Excellent
9	I/II	Excellent
10	II/III	Excellent
11	No finger involved	
12	II/III/IV	Excellent
13	I/V	Excellent
14	II	Good
	III	Excellent

I: thumb; II: index finger; III: middle finger; IV: ring finger; V: small finger.

## Data Availability

The datasets used and analysed during this study are available from the corresponding author on reasonable request.

## Abbreviations

ADM: Acellular dermal matrix
FTSG: Full-thickness skin graft
STSG: Split-thickness skin
TAM: Total active motion
VSD: Vacuum sealing drainage.

The article "Use of Composite Acellular Dermal Matrix-Ultrathin Split-Thickness Skin in Hand Hot-Crush Injuries: A One-Step Grafting Procedure" was retracted in 2023. Reasons: unreliable results or conclusions; concerns about the data; concerns about the peer review; concerns about the citations.

## References

[1] Sagi A., Amir A., Fliss D. M., Ozi S., Ofer G., Rosenberg L. (1997). Combined thermal and crush injury to the hand and fingers. *Burns*.

[2] Taras J. S., Sapienza A., Roach J. B., Taras J. P. (2010). Acellular dermal regeneration template for soft tissue reconstruction of the digits. *The Journal of Hand Surgery*.

[3] Reynolds M., Kelly D. A., Walker N. J., Crantford C., Defranzo A. J. (2018). Use of integra in the management of complex hand wounds from cancer resection and nonburn trauma. *Hand (N Y)*.

[4] Dast S., Vaucher R., Rotari V. (2017). Thin flaps in the management of hand and upper limb defects. *Annales de Chirurgie Plastique et Esthétique*.

[5] van der Veen V. C., van der Wal M. B., van Leeuwen M. C., Ulrich M. M., Middelkoop E. (2010). Biological background of dermal substitutes. *Burns*.

[6] Ellis C. V., Kulber D. A. (2012). Acellular dermal matrices in hand reconstruction. *Plastic and Reconstructive Surgery*.

[7] Teoh V., Gui G. (2020). Direct to implant breast reconstruction with biological acellular dermal matrices. *British Journal of Hospital Medicine*.

[8] Li X., Meng X., Wang X. (2015). Human acellular dermal matrix allograft: a randomized, controlled human trial for the long-term evaluation of patients with extensive burns. *Burns*.

[9] Hu Z., Zhu J., Cao X. (2016). Composite skin grafting with human acellular dermal matrix scaffold for treatment of diabetic foot ulcers: a randomized controlled trial. *Journal of the American College of Surgeons*.

[10] Chu C. S., McManus A. T., Matylevich N. P., Goodwin C. W., Pruitt B. A. (2002). Integra as a dermal replacement in a meshed composite skin graft in a rat model: a one-step operative procedure. *The Journal of Trauma*.

[11] Lee Y. J., Park M. C., Park D. H., Hahn H. M., Kim S. M., Lee I. J. (2017). Effectiveness of acellular dermal matrix on autologous split-thickness skin graft in treatment of deep tissue defect: esthetic subjective and objective evaluation. *Aesthetic Plastic Surgery*.

[12] Pan Y., Liang Z., Yuan S., Xu J., Wang J., Chen S. (2011). A long-term follow-up study of acellular dermal matrix with thin autograft in burns patients. *Annals of Plastic Surgery*.

[13] Kim Y. H., Hwang K. T., Kim K. H., Sung I. H., Kim S. W. (2019). Application of acellular human dermis and skin grafts for lower extremity reconstruction. *Journal of Wound Care*.

[14] Jeschke M. G., van Baar M. E., Choudhry M. A., Chung K. K., Gibran N. S., Logsetty S. (2020). Burn injury. *Nature Reviews Disease Primers*.

[15] Li Y., Li P. Y., Sun S. J. (2019). Chinese Trauma Surgeon Association for management guidelines of vacuum sealing drainage application in abdominal surgeries--update and systematic review. *Chinese Journal of Traumatology*.

The article "Use of Composite Acellular Dermal Matrix-Ultrathin Split-Thickness Skin in Hand Hot-Crush Injuries: A One-Step Grafting Procedure" was retracted in 2023. Reasons: unreliable results or conclusions; concerns about the data; concerns about the peer review; concerns about the citations.

[16] Libberecht K., Lafaire C., Van Hee R. (2006). Evaluation and functional assessment of flexor tendon repair in the hand. *Acta Chirurgica Belgica*.

[17] Di Castri A., Quarta L., Mataro I. (2018). The entity of thermal-crush-avulsion hand injury (hot–press roller burns) treated with fast acting debriding enzymes (nexobrid): literature review and report of first case. *Annals of burns and fire disasters*.

[18] Lewis R. E., Towery E. A., Bhat S. G. (2019). Human acellular dermal matrix is a viable alternative to autologous skin graft in patients with cutaneous malignancy. *The American Surgeon*.

[19] Lee M. C., Jang Y. J., Yun I. S., Lew D. H., Lee W. J. (2017). Comparative skin evaluation after split-thickness skin grafts using 2 different acellular dermal matrices to cover composite forearm defects. *The Journal of Hand Surgery*.

[20] Iorio M. L., Shuck J., Attinger C. E. (2012). Wound healing in the upper and lower extremities. *Plastic and Reconstructive Surgery*.

[21] Yi J. W., Kim J. K. (2015). Prospective randomized comparison of scar appearances between cograft of acellular dermal matrix with autologous split-thickness skin and autologous split-thickness skin graft alone for full-thickness skin defects of the extremities. *Plastic and Reconstructive Surgery*.

[22] Hicks K. E., Huynh M. N., Jeschke M., Malic C. (2019). Dermal regenerative matrix use in burn patients: A systematic review. *Journal of plastic, reconstructive & aesthetic surgery*.

[23] Maruccia M., Marannino P. C., Elia R. (2019). Treatment of finger degloving injury with acellular dermal matrices: functional and aesthetic results. *Journal of Plastic, Reconstructive & Aesthetic Surgery*.

[24] Kwa K. A. A., Goei H., Breederveld R. S., Middelkoop E., van der Vlies C. H., van Baar M. E. (2019). A systematic review on surgical and nonsurgical debridement techniques of burn wounds. *Journal of Plastic, Reconstructive & Aesthetic Surgery*.

[25] Yapici A. K., Kaldirim U., Arziman I., Ardic S., Eroglu M. (2016). Hot-press hand injury caused by roller type ironing machine. *Indian journal of plastic surgery*.

[26] Li Z., Wu W., Liu S., Hao Y. (2017). Effect of vacuum sealing drainage in dermatoplasty of large area of cutaneous defects. *International Journal of Surgery*.

